RETRACTED

# Clinical significance of the induction of macrophage differentiation by the costimulatory molecule B7-H3 in human non-small cell lung cancer

**DOI:** 10.3892/ol.2013.1586

**Published:** 2013-09-13

**Authors:** JING SUN, YONG MAO, YANG-QIN ZHANG, YUN-DI GUO, CHUAN-YONG MU, FENG-QING FU, XUE-GUANG ZHANG

**Affiliations:** 1 Institute of Medical Biotechnology, Suzhou Health College, Suzhou, Jiangsu 215009, P.R. China; 2 Department of Gastroenterology, The Fourth Affiliated Hospital of Soochow University, Wuxi, Jiangsu 214062, P.R. China; 3 Clinical Immunology Laboratory, The First Affiliated Hospital of Suzhou University, Suzhou, Jiangsu 215007, P.R. China

**Keywords:** non-small cell lung cancer, B7-H3, tumor-associated macrophage

## Abstract

B7-H3, a member of the B7 family of molecules, is expressed in certain types of human cancer and is important in tumor development and progression. Although several studies have reported that the expression of B7-H3 is correlated with poor outcomes in patients with cancer, its exact role in cancer remains unknown. In the present study, the expression levels of B7-H3 in the pathological specimens of 105 patients treated for non-small cell lung cancer (NSCLC) were examined by immunohistochemistry. A high expression level of B7-H3 was observed in 46.9% of the 105 NSCLC tissue specimens. These patients demonstrated a more advanced tumor grade and a shorter survival time. In addition, we also examined the levels of tumor-associated macrophages (TAMs) in NSCLC tissues and observed that the levels were positively correlated with the expression of B7-H3, and that higher levels of macrophages were associated with lower levels of infiltrating T cells and a shorter survival time. These results demonstrated that TAMs are important in the evasion of tumor immune surveillance in NSCLC. Furthermore, through knockdown of B7-H3 by RNA interference, we observed that soluble B7-H3 was capable of inducing macrophages to express higher levels of macrophage mannose receptor (MMR) and lower levels of human leukocyte antigen (HLA)-DR, as well as higher levels of interleukin-10 (IL-10) and lower levels of IL-1β *in vitro.* These observations are characteristic of an anti-inflammatory/reparatory (alternative/M2) phenotype. Therefore, our data suggests that B7-H3 proteins are involved in the progression of NSCLC by inducing the development of monocytes into anti-inflammatory cells.

## Introduction

Primary lung cancer is the leading cause of cancer-related mortality worldwide and has a poor prognosis compared with other types of cancer (1). Approximately 80% of all lung cancer cases are histologically classified as non-small cell lung cancer (NSCLC) (2). The overall 5-year survival rate of NSCLC is 10–15% (3), despite the availability of numerous treatment strategies, including conventional surgery, chemotherapy, radiotherapy, immunotherapy or a combination of these therapies (4). The pathogenesis of NSCLC involves multiple pathways and may result from numerous factors, such as smoking, bacterial infection and environmental contamination. Several studies have demonstrated that the overall survival and recurrence rates of lung cancer are associated with the type of local immune response (5).

RETRACTED

Macrophages are the primary immune cell type that infiltrates solid tumors, contributing ≤50% of the tumor cell mass (6). Consequently, these tumor-associated macrophages (TAMs) are important in determining the clinical outcome of disease. A number of studies have demonstrated that depending on the type of micro-environmental stimulation, TAMs are capable of exhibiting a pro-inflammatory (classical/M1) or an anti-inflammatory/reparatory (alternative/M2) phenotype (7–9). The M1 phenotype is known to suppress tumor growth, while the M2 phenotype promotes tumor growth. M1 macrophages are induced by lipopolysaccharide (LPS)/interferon-γ (IFN-γ) and are able to propagate the T helper 1 (Th1) response of T cells. Therefore, M1 macrophages are considered to be pro-inflammatory, which is reflected by their expression of interleukin-1β (IL-1β), IL-6, IL-8 or tumor necrosis factor-α (TNF-α). M2 macrophages are induced by IL-4 (M2a), immune complexes (M2b) or IL-13/IL-10 (M2c), and are mainly responsible for propagating the Th2 response of T cells. Thus, M2 macrophages are considered as anti-inflammatory, which is reflected by their expression of IL-10, CD36, scavenger receptor-A or the mannose receptor. Macrophages are critical in tumor progression; however, the mechanism by which the M2 phenotype is induced and promotes tumor angiogenesis is unclear.

B7-H3, a member of the B7 family, was cloned from a dendritic cell (DC) cDNA library in 2001 (10) and is expressed at low levels in several normal lymphoid and peripheral tissues (11). However, several studies have revealed that B7-H3 expression is elevated in numerous types of cancer, including lung cancer (12,13), prostate cancer (14,15), ovarian carcinoma (16), colorectal carcinoma (17), pancreatic cancer (18,19) and gastric cancer (20). These studies demonstrated a variety of conflicting functions for B7-H3; however, the majority of clinical data revealed a positive correlation between B7-H3 expression and tumor size, progression and prognosis. We hypothesize that the conflicting findings among different studies may be due to the existence of two isoforms of B7-H3: One of which is 4IgB7-H3, possessing four Ig-like domains in the extracellular domain; and the other of which is 2IgB7-H3, with two Ig-like domains in the extracellular domain due to alternative splicing (21,22). However, the expression patterns of each isoform in tumors and the mechanism by which the isoforms of B7-H3 affect cancer progression remain unknown.

RETRACTED

In the present study, the pathological specimens of 105 patients treated for NSCLC were evaluated by immunohistochemistry to characterize the expression levels of B7-H3 in human NSCLC tissues. A negative correlation between the expression levels of B7-H3 and the survival time of patients was observed. In addition, we identified an inverse correlation between B7-H3 expression and the levels of tumor-infiltrating macrophages, suggesting that B7-H3 is important in the suppression of tumor immune surveillance. Furthermore, we used *in vitro* assays to investigate the role of B7-H3 in regulating macrophage differentiation into M2 macrophages and its involvement in tumor progression. Taken together, our study establishes an important role of B7-H3 in cancer progression and suggests that the expression of B7-H3 may be involved in suppressing cancer immune surveillance.

## Materials and methods

### Patients

Tissues from 105 patients who underwent surgery for lung cancer between January and December, 2005 at the Department of Thoracic Surgery, The First Affiliated Hospital of Suzhou University (Suzhou, China) and The Fourth Affiliated Hospital of Soochow University (Wuxi, China) were used in the study. None of the patients received pre-operative chemotherapy or radiotherapy. The paraffin blocks of the tumor tissues were obtained from the archival collections of the Department of Pathology, The First Affiliated Hospital of Suzhou University and The Fourth Affiliated Hospital of Soochow University, and all 105 specimens were diagnosed with NSCLC by hematoxylin and eosin (H&E) staining. The patients’ pathological reports were reviewed and their clinical parameters are shown in Table I. This study was approved by the ethics committee of the First Affiliated Hospital of Suzhou University. Written informed consent was obtained from the patients.

### Cell culture and antibodies

The A549, H1299 and H460 lung cancer cell lines were purchased from the American Type Culture Collection (Manassas, VA, USA) and the SPCA-1 lung cancer cell line was purchased from the Shanghai Cell Biology Institute of the Chinese Academy of Sciences (Shanghai, China). The cells were cultured at 37ºC in a humidified incubator supplemented with 5% CO_2_. Peripheral blood mononuclear cells (PBMCs) were isolated by Ficoll-Hypaque gradient centrifugation from the peripheral blood of healthy donors (Suzhou Central Blood Bank, Suzhou, China). Mouse anti-human B7-H3 monoclonal antibody (clone no. 4H7) was established and characterized at the Clinical Immunology Laboratory, The First Affiliated Hospital of Suzhou University). Mouse anti-human CD3 monoclonal antibody (clone no. SP7), mouse anti-human CD68 monoclonal antibody (clone no. KP1) and horseradish peroxidase (HRP)-labeled goat anti-mouse/rabbit secondary antibody were purchased from Maixin Bio, Ltd. (Fuzhou, China). Macrophage mannose receptor (MMR; CD206) antibody labeled with FITC was purchased from BioLegend (San Diego, CA, USA) and human leukocyte antigen (HLA)-DR labeled with phycoerythrin was purchased from Immunotech (Marseille, France).

RETRACTED

### RT-PCR

RNA was extracted from the NSCLC cell lines and tissues using TRIzol reagent (Takara Bio, Inc., Shiga, Japan) and converted into cDNA with an oligo(dT) primer using the PrimeScript First Strand cDNA Synthesis kit (Takara Biomedical Technology, Dalian, China). The sequence of the sense primer used in the PCR was 5′-CACTGTGGTTCTGCCTCA-3′ and the sequence of the antisense primer was 5′-GCTGTCTTGGAGCCTTCT-3′. Both types of primers were synthesized by Invitrogen Life Technologies (Carlsbad, CA, USA).

### Western blotting for B7-H3

Western blot analysis was performed using standard protocols. NSCLC cell lines and tissues were acquired and lysed with RIPA lysis buffer (Beyotime, Nantong, China). The lysates were then run in reducing buffer on Tris-glycine 4–20% acrylamide gradient gels (Novex; Invitrogen Life Technologies) and transferred onto an Immobilon-P membrane (Millipore, Billerica, MA, USA). Mouse anti-human B7-H3 antibodies were used at a concentration of 1 μg/ml for 2 h. The membranes were washed three times with wash buffer prior to incubation with goat anti-mouse-HRP conjugate (Molecular Probes, Eugene, OR, USA) at 0.2 μg/ml for 1 h. The membranes were then developed by enhanced chemiluminescence (Amersham Biosciences, Pittsburg, PA, USA).

### Immunohistochemistry

Immunohistochemistry was performed using the Maixin-Bio™ method according to the manufacturer’s instructions. Briefly, 3-μm-thick consecutive sections were cut by a microtome, dewaxed in xylene and rehydrated through a series of graded ethanol solutions. Antigens were retrieved by heating the tissue sections at 100ºC for 30 min in citrate solution or EDTA solution when required. The sections were cooled down and immersed in 0.3% H_2_O_2_ solution for 20 min to block endogenous peroxidase activity, then rinsed in phosphate-buffered saline (PBS) for 5 min, blocked with 5% BSA at room temperature for 20 min, and incubated with primary antibodies against CD3, CD68 or B7-H3 (final concentration in use, 10 μg/ml) at 4ºC overnight. Negative controls were performed by replacing the specific primary antibody with PBS. Following three washes with PBS, the sections were incubated with secondary antibodies for 30 min at room temperature. Diaminobenzene was used as the chromogen and hematoxylin was used as the nuclear counterstain. The sections were dehydrated, cleared and mounted.

RETRACTED

### Evaluation of B7-H3 immunohistochemical staining

Two independent observers who were blinded to the clinicopathological parameters of the patients examined the immunohistochemically stained sections. The sections were considered as positive when the tumor cells demonstrated cytoplasmic or membranous B7-H3 immunostaining. The B7-H3 immunostaining intensities were scored according to the following scale: Grade 0, negative; grade 1, weak positive; grade 2, moderate positive and grade 3, strong positive. The negative grade represented no tumor cells demonstrating positive immunostaining. For the analysis, the B7-H3 immunostaining intensities were classified as follows: The sections scored as grades 0 and 1 were defined as the low expression group and the sections scored as grades 2 and 3 were defined as the high expression group.

### Evaluation of infiltrating T lymphocytes and macrophages in NSCLC tissues

Tumor infiltrating T lymphocytes and macrophages in the tumor nest were determined according to the immunostaining intensities of CD3 and CD68. Firstly, the infiltrating T lymphocytes and macrophages in the tumor stroma were examined at low magnification (×40) and categorized according to the densities as follows: Grade 0, scanty; grade 1, moderate infiltration; grade 2, abundant infiltration and grade 3, massive infiltration. The group containing grade 0 and 1 densities was defined as the low infiltration group and the group containing grade 2 and 3 densities was defined as the high infiltration group. The results from each of the five areas were averaged and used in the statistical analysis.

### Small interfering RNA (siRNA) experiments

Three stealth RNA interference (RNAi) and two control RNAi sequences were obtained from algorithms (Invitrogen Life Technologies) based against the sequence accession no. AJ583695 from GenBank. Stealth RNAi was pooled in equimolar amounts and used at a working concentration of 10 μM in order to knockdown B7-H3 expression. Control RNAi was also pooled in equimolar amounts and used at a working concentration of 10 μM. The SPCA-1 NSCLC cell line was transfected with RNAi using Lipofectamine™ 2000 (Invitrogen Life Technologies) and replated for 48 h prior to use. As an additional control, SPCA-1 cells were mock transfected without the use of RNAi. To evaluate the effect of transfection, real-time PCR was performed to analyze the levels of B7-H3 expression and the primer sequences used were as follows: 5′-GGCTGTCTGTCTGTCTCATTG-3′ and 5′-TCCATCATCTTCTTTGCTGTCA-3′ (Invitrogen Life Technologies).

RETRACTED

PBMCs were isolated by Ficoll-Hypaque gradient centrifugation from the peripheral blood of healthy donors (Suzhou Central Blood Bank). The CD14 Positive Selection kit (Stem Cell Therapeutics, Toronto, Ontario, Canada) was used to isolate human monocytes from PBMCs and the purity of the monocytes was >95%, as identified by anti-CD14 staining. Cell suspensions were added to flat-bottom 6-well plates at a density of 10^6^ cells/well and the plates were incubated at 37ºC and 5% CO_2_, with SPCA-1 cells (2.5×10^5^), which had been transfected with B7-H3-specific RNAi. To ensure there was cytokine secretion from tumor cells in the culture, the supernatant collected from the SPCA-1 cells was added and cultured for 7 days. The soluble B7-H3 in the supernatant does not interfere with the experimental results since the level of soluble B7-H3 in the SPCA-1 supernatant is extremely low. After 3 days, the cells were collected and incubated with MMR or HLA-DR for 30 min at 4ºC and washed. At the same time, the supernatants were harvested and frozen at −80ºC until assayed for the secretion of IL-10 and IL-1β (BD Biosciences, Franklin Lakes, NJ, USA).

### Statistical analysis

All data are expressed as the mean ± standard deviation. Statistical analysis was performed using the Student’s t-test and analysis of variance. Correlations were evaluated by the Pearson’s correlation test. P<0.05 was considered to indicate a statistically significant result.

## Results

### B7-H3 expression in NSCLC tissues and cell lines

In order to examine the B7-H3 expression levels in NSCLC tissues and cells, RT-PCR and western blotting were performed. We detected two unambiguous bands in the NSCLC tissues and cell lines. One predominant band at ~1500 bp represented the 4IgB7-H3 isoform and a minor band at ~800 bp represented the 2IgB7-H3 isoform (Fig. 1A). These data supported the results of several other studies conducted in normal tissues and cells (23,24). The expression of B7-H3 was regulated following RNA transcription (25) and the B7-H3 protein was only expressed in a minority of tissues and cells, including activated lymphocytes and tumor cells. To determine the protein expression levels of B7-H3, western blot analysis was performed and we observed that the two isoforms of B7-H3 were expressed equally in tumor tissues and cell lines (Fig. 1B). The band at 110 kDa represented the 4IgB7-H3 isoform and the band at ~65 kDa represented the 2IgB7-H3 isoform.

RETRACTED

We additionally characterized the expression of B7-H3 in resected specimens from 105 NSCLC patients by immunohistochemistry. Our results demonstrated that the intensity of B7-H3 expression varied and the immunolocalization of the B7-H3 molecule was predominantly in the membrane and cytoplasm of the tumor cells. We observed 58 cases of low B7-H3 expression, including 14 cases of grade 0 (Fig. 2A) and 44 cases of grade 1 (Fig. 2B). The other 47 cases were of high B7-H3 expression, including 33 cases of grade 2 (Fig. 2C) and 14 cases of grade 3 (Fig. 2D).

### Correlation of B7-H3 expression with the clinical parameters of patients

We analyzed B7-H3 expression in NSCLC tissues and observed that its expression had a positive correlation with a patient’s tumor grade (P=0.048), suggesting that B7-H3 is involved in cancer progression. However, the B7-H3 expression levels did not correlate with other clinicopathological parameters, including gender, age, tumor location, tumor size, nodal metastasis and distant metastasis (Table I).

We additionally examined whether there was an association between survival time and B7-H3 expression in tumor cells. The cumulative survival time was calculated using the Kaplan-Meier method and analyzed using the log-rank test. This analysis demonstrated that carcinoma patients with high B7-H3 expression exhibited significantly shorter survival times (P=0.0230; Fig. 3A).

### Infiltrating macrophages in NSCLC tissues and their correlation with B7-H3 expression, survival time and infiltrating T lymphocytes

Following the examination of the immunohistochemically stained sections, a mass of macrophages that had infiltrated NSCLC tissues was detected. To elucidate the underlying mechanisms participating in the effect of TAMs in NSCLC, we performed an immunohistochemical examination to detect the number of infiltrating macrophages labeled with CD68 and analyzed its correlation with survival time. The results demonstrated that a shorter survival time was associated with a higher number of infiltrating macrophages (Fig. 3B). To assess the signals by which B7-H3 regulates macrophage differentiation, we additionally examined whether there was an association between B7-H3 expression and TAMs. The infiltration of macrophages had a significant correlation with the expression of B7-H3. Tumor cells that expressed higher levels of B7-H3 exhibited higher levels of macrophage infiltration (Table II).

In order to assess whether the effect of TAMs was tumor-suppressive or tumor-facilitative, we examined the number of tumor-infiltrating T lymphocytes and its correlation with the number of TAMs in the specimens of 105 NSCLC patients by CD3 immunostaining. We observed that the level of T-cell infiltration in the tumor nest and stroma was correlated with nodal metastasis (P=0.042; Table I).

RETRACTED

### Function of B7-H3 in macrophage differentiation

To assess the role of B7-H3 in inducing the differentiation of macrophages, RNAi technology was used to knockdown B7-H3 expression in SPCA-1 cell lines prior to coculture with monocytes. Pools of specific or control RNAi were transfected into SPCA-1 cells and screened for effective inhibition of B7-H3. Effective and specific knockdown of B7-H3 persisted for at least 8 days following transfection and the highest rate of transfection was observed at 48 h.

Monocytes isolated from PBMCs were cocultured with SPCA-1 cells that had been transfected with pooled B7-H3 RNAi or pooled control RNAi, or with mock-transfected SPCA-1 (no RNAi) cells. After 3 days of coculture with B7-H3 knockdown SPCA-1 cells, the monocytes were harvested to assay the expression of MMR and HLA-DR. The monocytes cocultured with siB7-H3-treated SPCA-1 cells expressed lower MMR and higher HLA-DR levels compared with those cocultured with control RNAi-treated SPCA-1 cells (Fig. 4B and C). The production of IL-1β and IL-10 by macrophages was measured by enzyme-linked immunosorbent assay (ELISA). The monocytes cocultured with siB7-H3-treated SPCA-1 cells demonstrated increased levels of IL-1β cytokine production compared with those cocultured with SPCA-1 cells transfected with control RNAi (Fig. 5A). By contrast, the secretion of IL-10 by monocytes cocultured with siB7-H3-treated SPCA-1 cells was reduced compared with that of monocytes cocultured with SPCA-1 cells transfected with control RNAi FLS (Fig. 5B).

## Discussion

Although B7-H3 is a costimulatory molecule that is expressed in T cells, natural killer cells and antigen-presenting cells (11), its expression is not limited to immune cells. The B7-H3 protein is also expressed in osteoblasts (26), fibroblasts, fibroblast-like synoviocytes (24) and epithelial cells (27). This broad expression pattern most likely suggests that B7-H3 possesses more diverse immunological and nonimmunological functions, particularly in peripheral tissues. B7-H3 has been demonstrated to be highly expressed in a variety of different types of human cancer (28), including prostate cancer (15), gastric cancer (29), ovarian cancer (16), colorectal cancer (17) and urothelial cell carcinoma (30). The results of *in vitro* and *in vivo* studies strongly suggest a possible involvement of B7-H3 in the T-cell responses involved in the regulation of antitumor immunity (31,32), while the majority of other studies have proposed opposite functions for B7-H3. These studies have identified that higher levels of tumor B7-H3 expression were correlated with a more advanced tumor grade, more common lymph node metastasis, advanced pathological stage, shorter survival time and higher incidence of recurrence (33–35). In the present study, we demonstrated that B7-H3 was highly expressed in lung cancer cells. Increased B7-H3 expression was detected in 86.6% of the 105 NSCLC specimens examined. B7-H3 expression was significantly correlated with the patients’ survival time; higher levels of B7-H3 expression were associated with a shorter survival time. Based on previous studies and the results of the present study, we concluded that B7-H3 expression may play a critical physiological and pathological role in the oncogenesis and development of NSCLC; however, its exact role remains unclear.

RETRACTED

In the present study, we demonstrated that B7-H3 expression was positively associated with the levels of infiltrating macrophages and the number of macrophages had a negative correlation with the patients’ survival time. These data suggest that the macrophages that infiltrate the tumor tissues may be important in promoting tumor progression (7). TAMs exhibit a continuum of phenotypes ranging from pro-inflammatory (M1-like) to anti-inflammatory (M2-like), and these phenotypes vary in their effects on tumor cells. Furthermore, TAMs are considered as a polarized population of M2 macrophages, particularly when the tumor begins to invade, vascularize and develop (36,37). The classification of polarized macrophages, as either the M1 or M2 phenotype, is mainly based on the differential secretion of cytokines. The M1 phenotype secretes IL-12 and TNF-α, and the M2 phenotype secretes IL-10. Our present study demonstrated that the B7-H3 signal pathway significantly increased the levels of IL-10 secretion and MMR expression, consequently switching the macrophage phenotype from M1 to M2.

We have previously demonstrated that the soluble form of B7-H3 is released from monocytes, DCs and activated T cells, and is able to be detected using the ELISA assay established in the Clinical Immunology Laboratory, The First Affiliated Hospital of Suzhou University (38). In addition, we previously identified that the levels of soluble B7-H3 molecules in serum from patients with NSCLC or colorectal carcinoma were significantly higher compared with those in patients with other pulmonary diseases or healthy volunteers (17,39). A high level of circulating B7-H3 in patients was demonstrated to be correlated with node metastasis, distant metastasis and clinical stage. It was suggested that B7-H3 may provide a promising serum biomarker to improve NSCLC diagnosis and prognostic assessment (39). In the present study, we identified that soluble B7-H3 was only produced from the 2IgB7-H3 isoform, while the 4IgB7-H3 isoform was only expressed in the membrane (22). Thus, 2IgB7-H3 is highly expressed in tumor tissues as well as in tumor cell lines. However, the underlying mechanism of soluble B7-H3 in serum has yet to be elucidated. We hypothesize that soluble B7-H3 may function as a chemotactic factor, attracting monocytes in the peripheral blood to migrate to tumor tissues, inducing the development of macrophages, thereby promoting tumor oncogenesis and development.

RETRACTED

In conclusion, our present study indicated that the costimulatory molecule B7-H3 is important in NSCLC progression. The significantly elevated levels of soluble B7-H3 were stimulated by highly expressed 2IgB7-H3 on tumor cells. The B7-H3 signaling pathway may be involved in switching macrophages to the M2 phenotype and the negative regulation of the T lymphocyte-mediated immune response. Future studies should focus on examining the precise mechanism by which B7-H3 expression is regulated in the tumor environment. Overall knowledge of the clinical implications of this and of potential therapeutic interventions targeting the B7-H3 signaling pathway in NSCLC warrant further investigation.

## Figures and Tables

**Figure 1:** Expression of B7-H3 in lung cancer cell lines and tumor tissues. (A) PCR analysis of the A549, H460, H1299 and SPCA-1 lung cancer cell lines and tumor tissues using a B7-H3-specific primer. PCR analysis was performed in over six cases of non-small cell lung cancer. The product of ~1500 bp corresponded with the 4IgB7-H3 molecule, whereas the product of 800 bp corresponded with the 2IgB7-H3 gene. (B) Identification of B7-H3 isoforms in the lung cancer cell lines and tumor tissues. The membrane proteins extracted from the A549, H460, H1299 and SPCA-1 cell lines, and tumor tissues were detected by western blotting using a B7-H3 antibody. A band of ~110 kDa represented the 4IgB7-H3 protein, while a protein of ~65 kDa represented the 2IgB7-H3 protein.

**Figure 2:** B7-H3 immunostaining in non-small cell lung cancer tissues. (A) Negative, (B) weak positive, (C) moderate positive and (D) strong positive. Magnification, ×400. Diaminobenzene was used as the chromogen and hematoxylin was used as the nuclear counterstain.

**Figure 3:** Kaplan-Meier survival analysis of the correlation between survival time and the expression of B7-H3 or the number of infiltrating macrophages labeled with CD68 in 36 patients with non-small cell lung cancer.

RETRACTED

**Figure 4:** B7-H3 may inhibit the differentiation of monocytes into TAMs in the SPCA-1 cell line. (A) SPCA-1 cell lines highly express B7-H3. (B) Monocytes may express higher levels of MMR and lower levels of HLA-DR when cocultured with the SPCA-1 cell line. (C) Monocytes were cocultured with SPCA-1 cells transfected with pooled B7-H3-specific RNAi. SPCA-1 cells lose the ability to induce the differentiation of monocytes when transfected with B7-H3-specific RNAi. TAMs, tumor-associated macrophages; MMR, macrophage mannose receptor; HLA, human leukocyte antigen.

**Figure 5:** Monocytes were harvested following 3 days of coculture with SPCA-1 cells. The cytokine levels in the supernatants were measured by enzyme-linked immunosorbent assay. Error bars represent 95% confidence intervals. The two-tailed t-test analysis was used to compare cytokine production from monocytes cultured with SPCA-1 or SPCA-1 (RNAi). (A) IL-10 and (B) IL-1β production. The data are representative of three experiments with pooled B7-H3 RNAi or pooled control RNAi (control). IL, interleukin; RNAi, RNA interference.

**Table I:** Correlation between clinical parameters, B7-H3 expression and T-cell infiltration.

		B7-H3 expression			Macrophage infiltration			T-cell infiltration		
				
Clinical parameter	Cases	Low	High	P-value^a^	Low	High	P-value	Low	High	P-value
Gender										
Male	77	43 (42.5)^b^	34 (34.4)	0.835	39 (43.2)	38 (32.7)	0.094	36 (38.9)	41 (38.1)	0.206
Female	28	15 (15.5)	13 (12.5)		20 (15.7)	8 (12.3)		17 (14.1)	11 (13.9)	
Age (years)										
≤60	51	28 (28.2)	23 (22.8)	0.946	29 (28.7)	22 (22.3)	0.893	27 (25.7)	24 (25.2)	0.624
>60	54	30 (29.8)	24 (24.1)		30 (30.3)	24 (23.7)		26 (27.3)	28 (26.7)	
Histological subtype										
Adenocarcinoma	45	26 (24.9)	19 (20.1)	0.720	24 (28.2)	21 (26.8)	0.023^e^	22 (22.7)	23 (22.3)	0.869
Squamous cell carcinoma	47	24 (26.0)	23 (21.0)		31 (24.1)	16 (22.9)		25 (23.7)	22 (23.3)	
Large cell carcinoma	13	8 (7.2)	5 (5.8)		4 (6.37)	9 (6.3)		6 (6.6)	7 (6.4)	
Tumor size (cm)										
≤4	54	32 (29.8)	22 (24.2)	0.393	32 (30.3)	22 (22.7)	0.514	25 (27.3)	29 (26.7)	0.378
>4	51	26 (28.2)	25 (22.8)		27 (28.7)	24 (22.3)		28 (25.7)	23 (25.2)	
Tumor status^c^										
pT1	11	8 (7.6)	3 (2.8)	0.048^e^	7 (7.4)	4 (5.6)	0.302	4 (6.6)	7 (6.4)	0.618
pT2	45	30 (28.6)	15 (14.3)		28 (25.2)	17 (20.8)		22 (24.7)	23 (24.3)	
pT3	31	13 (12.4)	18 (17.1)		13 (15.3)	18 (11.7)		18 (13.6)	13 (13.4)	
pT4	18	7 (6.7)	11 (10.5)		11 (9.1)	7 (2.9)		10 (8.1)	8 (7.9)	
Nodal metastasis										
Without	47	26 (26.0)	21 (21.0)	0.988	29 (26.3)	18 (20.7)	0.305	19 (24.1)	28 (22.8)	0.042^e^
With	58	32 (32.0)	26 (26.0)		30 (31.8)	28 (25.2)		35 (29.8)	23 (28.1)	
Distant metastasis^d^										
Without	101	56 (55.8)	45 (45.2)	0.765	59 (56.2)	42 (42.8)	0.072	50 (51.0)	51 (50.0)	0.624
With	4	2 (2.21)	2 (1.79)		0 (2.8)	4 (2.2)		3 (2.02)	1 (1.98)	

a P-values were calculated using the Pearson’s χ^2^ test or the χ^2^ test for trend.

b Numbers inside the parentheses represent the percentage of patients.

c The stage was determined by pathological (p) examination. T1, tumor ≤3 cm diameter, surrounded by lung or visceral pleura, without invasion and more proximal than the lobar bronchus. T2, tumor >3 cm, however ≤7 cm, or a tumor with any of the following features: Involvement of the main bronchus >2 cm distal to the carina; invasion of the visceral pleura; association with atelectasis or obstructive pneumonitis that extends to the hilar region, however, does not involve the entire lung. T3, tumor >7 cm diameter or with any of the following features: Direct invasion of the chest wall, diaphragm, phrenic nerve, mediastinal pleura, parietal pericardium or main bronchus <2 cm from the carina without involvement of the carina; atelectasis or obstructive pneumonitis of the entire lung or separate tumor nodules in the same lobe. T4, tumor of any size that invades the mediastinum, heart, great vessels, trachea, recurrent laryngeal nerve, esophagus, vertebral body and carina, or with separate tumor nodules in a different ipsilateral lobe.

d These patients demonstrated distant metastasis, and presented with metastais of the brain or bone.

e Signifies P<0.05.

RETRACTED

**Table II:** Correlation between the levels of infiltrating macrophages and B7-H3 expression or T lymphocytes in NSCLC tissues.

	Infiltrating macrophages in NSCLC tissues					
			
Group	Low (n)	Ratio (%)	High (n)	Ratio (%)	χ^2^ value	P-value
B7-H3 expression	59	56.19	46	43.80	4.5788	0.0324^a^
Low expression	38	36.19	20	19.04		
High expression	21	20.00	26	24.76		
Infiltrating T lymphocytes	59	56.19	46	43.81	4.9567	0.0260^a^
Low infiltrating	36	34.29	18	17.14		
High infiltrating	23	21.90	28	26.67		
Total	105		105			

a Signifies P<0.05.

NSCLC, non-small cell lung cancer; n, number of cases.

## References

[1] Patrick DJ, Fitzgerald SD, Sesterhenn IA, Davis CJ, Kiupel M (2006). Classification of canine urinary bladder urothelial tumours based on the World Health Organization/International Society of Urological Pathology consensus classification. J Comp Pathol.

[2] Gansler T, Ganz PA, Grant M (2011). Sixty years of CA: a cancer journal for clinicians. CA Cancer J Clin.

[3] Ginsberg RJ (1997). Resection of non-small cell lung cancer: how much and by what route. Chest.

[4] Payne DG (1993). The role of radiotherapy in bronchopulmonary cancer. Rev Mal Respir.

[5] Derniame S, Vignaud JM, Faure GC, Béné MC (2008). Alteration of the immunological synapse in lung cancer: a microenvironmental approach. Clin Exp Immunol.

RETRACTED

[6] Faget J, Biota C, Bachelot T (2011). Early detection of tumor cells by innate immune cells leads to T(reg) recruitment through CCL22 production by tumor cells. Cancer Res.

[7] Mantovani A, Bottazzi B, Colotta F, Sozzani S, Ruco L (1992). The origin and function of tumor-associated macrophages. Immunol Today.

[8] Mantovani A, Allavena P, Sica A (2004). Tumour-associated macrophages as a prototypic type II polarised phagocyte population: role in tumour progression. Eur J Cancer.

[9] Mantovani A, Sozzani S, Locati M (2004). Infiltration of tumours by macrophages and dendritic cells: tumour-associated macrophages as a paradigm for polarized M2 mononuclear phagocytes. Novartis Found Symp.

[10] Chapoval AI, Ni J, Lau JS (2001). B7-H3: a costimulatory molecule for T cell activation and IFN-gamma production. Nat Immunol.

[11] Sun M, Richards S, Prasad DV, Mai XM, Rudensky A, Dong C (2002). Characterization of mouse and human B7-H3 genes. J Immunol.

[12] Sun Y, Liu J, Gao P, Wang Y, Liu C (2008). Expression of Ig-like transcript 4 inhibitory receptor in human non-small cell lung cancer. Chest.

[13] Sun Y, Wang Y, Zhao J (2006). B7-H3 and B7-H4 expression in non-small-cell lung cancer. Lung Cancer.

[14] Chavin G, Sheinin Y, Crispen PL (2009). Expression of immunosuppresive B7-H3 ligand by hormone-treated prostate cancer tumors and metastases. Clin Cancer Res.

[15] Lehmann BD, Paine MS, Brooks AM (2008). Senescence-associated exosome release from human prostate cancer cells. Cancer Res.

[16] Zang X, Sullivan PS, Soslow RA (2010). Tumor associated endothelial expression of B7-H3 predicts survival in ovarian carcinomas. Mod Pathol.

[17] Sun J, Chen LJ, Zhang GB (2010). Clinical significance and regulation of the costimulatory molecule B7-H3 in human colorectal carcinoma. Cancer Immunol Immunother.

[18] Yamato I, Sho M, Nomi T (2009). Clinical importance of B7-H3 expression in human pancreatic cancer. Br J Cancer.

[19] Loos M, Hedderich DM, Ottenhausen M (2009). Expression of the costimulatory molecule B7-H3 is associated with prolonged survival in human pancreatic cancer. BMC Cancer.

[20] Wu CP, Jiang JT, Tan M (2006). Relationship between co-stimulatory molecule B7-H3 expression and gastric carcinoma histology and prognosis. World J Gastroenterol.

[21] Ling V, Wu PW, Spaulding V (2003). Duplication of primate and rodent B7-H3 immunoglobulin V- and C-like domains: divergent history of functional redundancy and exon loss. Genomics.

[22] Sun J, Fu F, Gu W (2011). Origination of new immunological functions in the costimulatory molecule B7-H3: the role of exon duplication in evolution of the immune system. PLoS One.

RETRACTED

[23] Zhou YH, Chen YJ, Ma ZY (2007). 4IgB7-H3 is the major isoform expressed on immunocytes as well as malignant cells. Tissue Antigens.

[24] Tran CN, Thacker SG, Louie DM (2008). Interactions of T cells with fibroblast-like synoviocytes: role of the B7 family costimulatory ligand B7-H3. J Immunol.

[25] Xu H, Cheung IY, Guo HF, Cheung NK (2009). MicroRNA miR-29 modulates expression of immunoinhibitory molecule B7-H3: potential implications for immune based therapy of human solid tumors. Cancer Res.

[26] Suh WK, Wang SX, Jheon AH (2004). The immune regulatory protein B7-H3 promotes osteoblast differentiation and bone mineralization. Proc Natl Acad Sci USA.

[27] Saatian B, Yu XY, Lane AP (2004). Expression of genes for B7-H3 and other T cell ligands by nasal epithelial cells during differentiation and activation. Am J Physiol Lung Cell Mol Physiol.

[28] Chen YW, Tekle C, Fodstad O (2008). The immunoregulatory protein human B7H3 is a tumor-associated antigen that regulates tumor cell migration and invasion. Curr Cancer Drug Targets.

[29] Arigami T, Uenosono Y, Hirata M, Yanagita S, Ishigami S, Natsugoe S (2011). B7-H3 expression in gastric cancer: a novel molecular blood marker for detecting circulating tumor cells. Cancer Sci.

[30] Boorjian SA, Sheinin Y, Crispen PL (2008). T-cell coregulatory molecule expression in urothelial cell carcinoma: clinicopathologic correlations and association with survival. Clin Cancer Res.

[31] Kobori H, Hashiguchi M, Piao J, Kato M, Ritprajak P, Azuma M (2010). Enhancement of effector CD8+ T-cell function by tumour-associated B7-H3 and modulation of its counter-receptor triggering receptor expressed on myeloid cell-like transcript 2 at tumour sites. Immunology.

[32] Loos M, Hedderich DM, Friess H, Kleeff J (2010). B7-h3 and its role in antitumor immunity. Clin Dev Immunol.

[33] Crispen PL, Sheinin Y, Roth TJ (2008). Tumor cell and tumor vasculature expression of B7-H3 predict survival in clear cell renal cell carcinoma. Clin Cancer Res.

[34] Hofmeyer KA, Ray A, Zang X (2008). The contrasting role of B7-H3. Proc Natl Acad Sci USA.

[35] Katayama A, Takahara M, Kishibe K (2011). Expression of B7-H3 in hypopharyngeal squamous cell carcinoma as a predictive indicator for tumor metastasis and prognosis. Int J Oncol.

[36] Mantovani A, Sozzani S, Locati M, Allavena P, Sica A (2002). Macrophage polarization: tumor-associated macrophages as a paradigm for polarized M2 mononuclear phagocytes. Trends Immunol.

[37] Murdoch C, Muthana M, Coffelt SB, Lewis CE (2008). The role of myeloid cells in the promotion of tumour angiogenesis. Nat Rev Cancer.

RETRACTED

[38] Zhang G, Hou J, Shi J, Yu G, Lu B, Zhang X (2008). Soluble CD276 (B7-H3) is released from monocytes, dendritic cells and activated T cells and is detectable in normal human serum. Immunology.

[39] Zhang G, Xu Y, Lu X (2009). Diagnosis value of serum B7-H3 expression in non-small cell lung cancer. Lung Cancer.

